# Circular RNA SOX13 promotes malignant behavior and cisplatin resistance in non-small cell lung cancer through targeting microRNA-3194-3p/microtubule-associated protein RP/EB family member 1

**DOI:** 10.1080/21655979.2021.1997223

**Published:** 2022-01-11

**Authors:** Libin Zhang, Hao Peng, Zheyuan Xu, Qiuju Yang, Yang Wang, Han Wang, Liang Bu

**Affiliations:** a Department of Thoracic Surgery, The First People’s Hospital of Yunnan Province, Kunming City, Yunnan Province, China; b Department of Thoracic Surgery, Kunming University of Science and Technology, School of Medicine, Kunming City, Yunnan Province, China

**Keywords:** CircSOX13, mir-3194-3p, marep1, cisplatin resistance, non-small cell lung cancer

## Abstract

Circular RNA (circRNA) presents an essential regulatory role in affecting the occurrence and acquired resistance in non-small cell lung cancer (NSCLC), but how circSOX13 impacts NSCLC is unclear. In this work it was found that compared with adjacent normal tissues, circSOX13 and the microtubule-associated protein RP/EB family member 1 (MAPRE1) were signally up-regulated in NSCLC while miR-3194-3p was signally lowered. Pulmonary function tests (PETs) revealed that knocking down circSOX13 or overexpressing miR-3194-3p inhibited NSCLC proliferation, invasion and migration but promoted its apoptosis. The promoting effect of overexpressing circSOX13 on NSCLC was reversed via knocking down MAPRE1. Additionally, knocking down circSOX13 reduced cisplatin resistance in NSCLC. Furthermore, circSOX13 mediated MAPRE1 expression via competitively binding miR-3194-3p to exert its tumorigenic impact. To conclude, this work clarified the carcinogenic impact of circSOX13-miR-3194-3p-MAPRE1 axis on NSCLC and DDP resistance. CircSOX13 can be a potential diagnostic marker and therapeutic target for NSCLC, thus providing a new insight for clinically reversing its acquired resistance.

## 1 Introduction

Lung cancer, a universal cancer, features the highest incidence and mortality worldwide [1,2]. Among various lung cancers, the most common is non-small cell lung cancer (NSCLC), taking up about 80% [3]. NSCLC is allocated into three different subtypes, including squamous cell carcinoma, adenocarcinoma and large cell lung carcinoma [4]. Treating NSCLC mainly relies on surgical resection and chemotherapy or radiation therapy [5,6]. However, due to the acquired resistance, the clinical effect and prognosis of NSCLC are still poor [7,8]. Therefore, further understanding the potential molecular mechanisms of NSCLC malignant behavior and resistance is very vital for improving the prognosis.

Circular RNA (circRNA), an endogenous, covalently blocked RNA, is abundantly expressed in tissues with stability [9,10]. More and more studies have revealed that circRNA functions as an essential role in various malignant behaviors of NSCLC. Recently, Li N *et al*. found that circ_0017956 can promote NSCLC proliferation and metastasis via regulating the miR-515-5p/Integrin Beta 8 (ITGB8) axis [11]. In addition, studies have shown that circRNA hsa_circ_0072309 promotes tumorigenesis and invasion via regulating the miR-607/FTO axis in NSCLC [12]. CircRNA is also involved in regulating the chemoresistance or radiosensitivity in NSCLC. Based on the latest research, silencing circPVT1 enhances the radiosensitivity in NSCLC via regulating microRNA(miRNA)-1208 [13]. Another study revealed that circRNA_100565 facilitates cisplatin-resistant NSCLC via adjusting miR-337-3p/a disintegrin and metalloproteinases 28 (ADAM28) axis in proliferation, apoptosis and autophagy [14]. CircSOX13 is a type of circRNA. Based on a recent study, circSOX13 is differentially expressed in NSCLC [15]. However, whether it affects the malignant behavior and cisplatin resistance in NSCLC is unclear.

In this work, it was intended to determine the role circSOX13 playing in the malignant behavior and cisplatin resistance in NSCLC, finding that high-expression circSOX13 promotes them. These effects of circSOX13 mainly rely on crosstalk with miR-3194-3p and microtubule-associated protein RP/EB family member 1 (MAPRE1).

## 2. Methods

### 2.1 Clinical samples

From 2014 to 2017, 54-pair NSCLC and adjacent normal tissue were accessed from patients undergoing surgery in the first people’s Hospital of Yunnan Province but not receiving chemotherapy or radiation therapy. Blood samples were collected from 14 healthy subjects who came to our hospital for physical examination and 31 NSCLC patients for treatment. The serum was obtained via centrifugation at 1,500 rpm for 15 min., Based on the clinicopathological diagnosis of pathology department, all subjects were diagnosed as NSCLC. Their detailed follow-up data on clinicopathological characteristics were accessed. This study has got the Ethics board approval of the first people’s Hospital of Yunnan Province with all patients’ written informed consent. Serum and tissue samples were stored at −80°C immediately after sampling until RNA or protein were extracted.

### 2.2 Cell culture

Normal human bronchial epithelial cell line (16HBE) and parental NSCLC cell lines (PC9, SPC-A1, H1975, H1299 and A549) were bought from ATCC and placed in incubators under at 37°C with 5% CO_2_. The above cells identified by Abace Biotechnology were confirmed to be mycoplasma-free. Parental NSCLC cells were received with culture in Gibco RPMI-1640 medium containing 10% Fetal bovine serum (FBS); 16HBE cells were cultured in Dulbecco’s Modified Eagle Medium (Invitrogen, Carlsbad, California, USA) . To induce cisplatin resistance in NSCLC cells (DDP/NSCLC), these cells were received with 80-d exposure to continuous low-dose cisplatin (0.5 μg/mL-5 μg/mL, Sigma-Aldrich, Shanghai, China).

### 2.3 Cell transfection

The overexpression vector of circRNA SOX13 (oe-SOX13) and negative control (oe-NC) were designed and constructed by Vazamy (China). Short harpin RNA targeting circRNA SOX13 (sh-SOX13), short hairpin RNA NC (sh-NC), small interfering RNA targeting MAPRE1 (si-MAPRE1), small interfering RNA NC (si-NC), miR-3194-3p mimic/inhibitor and mimic/inhibitor NC were purchased from Sangon Biotech (Shanghai, China). The above vectors were delivered to NSCLC cells or DDP/NSCLC cells using Lipofectamine 2000 reagent (Invitrogen, CA, USA) according to the manufacturer’s protocol. After 48 h, the cells were collected for subsequent experiments, and the transfection efficiency was verified by reverse transcription quantitative polymerase chain reaction (RT-qPCR).,

### 2.4 Cell counting kit (CCK)-8 to detect cell viability or IC_50_ value

In IC_50_ analysis, A549/DDP and H1299/DDP cells were received with implantation into 96-well plates overnight, later exposed to different concentrations of DDP (10, 20, 40, 60, 80, and 100 μM) for 48 hours [16]. After 10 μL of CCK-8 solution (Dojindo, Kumamoto, Japan) was supplemented to every well, the cultured things were received with incubation for another 4 hours at 37°C. Via enzyme-labeled instruments the optical density was recorded at 450 nm. The calculation of IC_50_ value was done based on the dose-response survival curve. With cell viability determination, the transfected cells were added to 96-well plates for growth, 10 μL of CCK-8 solution was supplemented at 0, 24, 48, 72 and 96 h, and the optical density measured at 450 nm was done after 4-hour incubation. The experiment was carried out 3 times.

### 2.5 Flow cytometry

In reference to manufacturer’s protocol, cell apoptosis was checked via BD Bioscience AV- fluoresceinisothiocyanat (FITC)/propidium iodide (PI) Apoptosis Detection Kit [17]. The cells were subject to staining with AV-FITC/PI in the dark for 35 minutes at room temperature. Later, the apoptosis rate was measured via flow cytometers (FCM, Thermo Fisher Scientific, U.S.).

### 2.6 Transwell

Via Transwell chamber (pore size of 8 μm, Corning) without matrigel (migration) or matrigel coating (invasion) (Bection Dickinson, U.S.) the cell migration and invasion abilities were measured. Then transfected cells (2 × 10^4^ cells) were implanted into upper chambers; 500 μL of culture medium with 10% FBS was applied as a chemoattractant to place into lower chambers. Transwell system was kept at 37°C for 24 hours. After cell removal on the top surface with cotton swabs, the cells on the bottom were received with 15-minute staining with 0.1% crystal violet at room temperature, and later were photographed and counted in five predetermined fields of view (×200). The experiment was repeated three times.

### 2.7 Dual luciferase reporter (DLR) experiment

Full-length circRNA SOX13 and MAPRE1 3ʹuntranslated region (UTR) was inserted into Promega pGL4 luciferase reporter vectors, thereby establishing wild-type circRNA SOX13 (circRNA SOX13-WT) and MAPREl (MAPRE1-WT) vectors. Later, the putative binding sites of miR-3194-3p in circRNA SOX13 and MAPRI1 3ʹUTR were given mutation to establish their mutant (MUT) vectors (circRNA SOX13-MUT and MAPRE1-MUT). A549 and H1299 cells (5 × 10^4^/well) done with passage in 24-well plates. Later, the above-mentioned vectors (300 ng) were received with co-transfection with miR-3194-3p mimic/NC (10 μM) via Lipofectamine 2000 reagent (Invitrogen) into cells. After 48 h, the luciferase activity was given detection via Promega DLR system.

### 2.8 RT-qPCR

In reference to manufacturer’s instructions, via TRIzol reagent (Invitrogen, U.S.) total RNA extraction from tissues or cells was done. PrimeScript RT kit (TaKaRa) was utilized to reversely transcribe total RNA (500 ng) into cDNA (10 μL). SYBR Premix Ex Taq (Takara) was applied to quantify mRNA in a real-time detection system (ABI7500), as well as Bulge-Loop miRNA qRT-PCR primer kit (RiboBio) to determine miRNA concentration, glyceraldehyde-3-phosphate dehydrogenase (GAPDH) and U6 as the quantification standardization of mRNA and miRNA, respectively. The 2^−ΔΔCt^ method was utilized to count gene expression. The primer sequence was detailed in Table 1.

**Table 1.** RT-qPCR primer sequences

	Primer sequences (5′ – 3′)
GAPDH	Forward: 5ʹ-CCTCGTCTCATAGACAAGATGGT-3’
	Reverse: 5ʹ-GGGTAGAGTCATACTGGAACATG-3’
U6	Forward: 5ʹ-CTCGCTTCGGCAGCACA-3’
	Reverse: 5ʹ-AACGCTTCACGAATTTGCGT-3’
CircSOX13	Forward: 5ʹ- AGTGATGTGGCCCCTACA AG-3’
	Reverse: 5ʹ- CCACTGGAGACCACTGGTTG −3’
MiR-3194-3p	Forward: 5ʹ- TCGGCAGGUCUGGCUCCGUGUC −3’
	Reverse: 5ʹ- CCGAGGACGGGAGTG −3’

### 2.9 Western blot

Total protein extraction from tissues and cell lines was implemented in Radio-Immunoprecipitation assay reagent (Beyotime Biotechnology Co., Ltd., Shanghai, China) with protease inhibitor phenylmethylsulfonyl fluoride (Sigma-Aldrich). The protein sample (20 μg) at the same amount was separated via sulfate polyacrylamide gel electrophoresis, and transferred to Polyvinylidene fluoride films (Millipore Corporation, Billerica, Massachusetts, USA) [18]. After blocking in 5% skimmed milk, the films were received with incubation with the following primary antibodies (Abcam Inc., Cambridge, MA, USA): MAPRE1 (ab50188), GAPDH (ab8245) at 4°C overnight. After wash with phosphate buffer saline (PBS) buffer for 3 times at room temperature, the films were received with incubation with secondary antibody (Abcam) for 120 minutes. At last, the protein bands were received with visualization on electrogenerated chemiluminescence system (GE Healthcare Bio-science, U.S.) and quantification was via Image J software with GAPDH as an internal reference.

### 2.10 Edu analysis

The proliferating cells were received with evaluation based on the protocol of EdU labeling/detection kit (Ribobio, Guangzhou, China). The cells were received with a 2-d culture in 12-well plates (5 × 10^4^ cells/well). Next, the cells were transferred to 50 μM EdU-labeled medium to culture in a standard incubator for 2 hours. The cultured cells were received with treatment with 4% paraformaldehyde (pH 7.4) for 30 minutes at room temperature, and later with 0.5% Triton X-100 for 20 minutes. After wash with PBS, the sample was stained with anti-EdU working solution for 30 minutes without luminescence at room temperature, with 4ʹ,6-dimidyl-2-phenylindole (DAPI) as a nuclear/chromosome counterstain. Cell observation was done via fluorescence microscopes. EdU positive cells was calculated from five random fields in three wells.

### 2.11 Tumor xenograft

Thirty 4-week-old male BALB/c nude mice were collected from Hunan SJA Laboratory Animal Co., Ltd. (Changsha, China) and kept in a specific pathogen-free animal facility on a 12-h light cycle with eating and drinking at will. After one week of adaptive feeding, A549 cells stably expressing sh-NC and sh-circSOX13 were subcutaneously injected into nude mice through the armpit of the right forelimb. The DDP group was injected with DDP twice a week (5 mg/kg) and the other groups were injected with the same dose of normal saline for 4 weeks when obvious tumors appeared. A vernier caliper was used to calculate the tumor length diameter (a) and short diameter (b) on a weekly basis to assess tumor volume. The volume formula was: a × b^2^ × 0.5. Four weeks later, the nude mice were euthanized, and the tumor tissues were collected, weighed and stored at −80°C for subsequent Western blot analysis. The animal experiment program was approved by the Animal Experiment Ethics Committee of XXXX Hospital. All animal procedures followed the guidelines for the Care and Use of Laboratory Animals published by the National Institutes of Health in Bethesda, Maryland, USA.

### 2.12 Statistics

Statistical analysis was done via SPSS 21.0 (SPSS Inc, U.S.) and detailed in mean ± standard deviation (SD). Student’s t test was applied for intergroup comparison, whereas one-way analysis of variance (ANOVA) was for comparisons among multiple groups. It was statistically significant at P*<0.05.

## 3 Results

### 3.1 Elevated circSOX13 is in NSCLC

Based on previous studies, circSOX13 was highly expressed in NSCLC tissues. In this study circSOX13 expression was further checked in NSCLC, which was signally higher than that in normal tissues adjacent to cancer (Figure 1a); In addition, serum circSOX13 was clearly elevated in NSCLC patients versus normal subjects (Figure 1b). In five NSCLC cell lines it was also visually higher than that of 16HBE (Figure 1c). Next, in the work it was examined the correlation between circSOX13 and NSCLC clinicopathological characteristics. According to the median circSOX13 expression in NSCLC, NSCLC patients were allocated into circSOX13 high expression group and circSOX13 low expression group. Higher CircSOX13 levels were visually linked with TNM stage and lymph node metastasis in NSCLC (Table 2).

**Table 2.** Correlation between circSOX13 and clinicopathological characteristics

Characteristics	Groups	Cases	CircSOX13 expression level		*P*
			High expression group (n = 27)	Low expression group (n = 27)	
Age	< 55	19	11	8	0.3926
	55 or more	35	16	19	
Gender	Male	39	17	22	0.1287
	Female	15	10	5	
Tumor size (cm)	<5 cm	21	13	8	0.1628
	5 cm or more	33	14	19	
Lymph node metastasis	Yes	37	24	13	0.0013
	No	17	3	14	
History of smoking	Yes	32	13	19	0.0966
	No	22	14	8

**Figure 1.** **CircSOX13 is highly expressed in NSCLC**. A. RT-qPCR to detect circSOX13 expression in NSCLC tissues and normal tissues adjacent to cancer; B. RT-qPCR to detect circSOX13 expression in serum of normal subjects and patients with NSCLC; C. RT-qPCR to detectcircSOX13 expression in PC9, SPC-A1, H1975, H1299 and A549 and 16HBE; the values were expressed by mean ± SD (C, n = 3); versus the normal tissue group, * *P* < 0.05; versus the 16HBE group,^ *P* < 0.05.

### 3.2 CircSOX13 knockdown represses NSCLC proliferation, migration, invasion and apoptosis

Next, in the work it was examined the impact of circSOX13 on the malignant behavior of NSCLC. A549 and H1299 with the highest circSOX13 expression were selected for follow-up experiments. The shRNA targeting circSOX13 was transfected to knock down circSOX13 in A549 and H1299 where circSOX13 expression was signally reduced after transfection (Figure 2a). CCK-8 and Edu analysis revealed that knocking down circSOX13 signally reduced the cell viability and proliferation rate of A549 and H1299 (Figures 2B and Figures 2C). Flow cytometry findings revealed that knocking down circSOX13 promoted A549 and H1299 apoptosis rate (Figure 2d). Later, in Transwell the invasion and migration capabilities of NSCLC were further checked, finding that knocking down circSOX13 signally reduced A549 and H1299 invasion and migration abilities (Figure 2e). These findings imply that knocking down circSOX13 prevents the malignant behavior.

**Figure 2.** **Knocking down circSOX13 inhibits NSCLC proliferation, migration and invasion but promotes apoptosis**. After transfecting circSOX13-shRNA, A. RT-qPCR to detect circSOX13 expression in A549 and H1299; B. CCK-8 to detect the viability of A549 and H1299; C. Edu analysis to detect A549 and H1299 proliferation cell; D. Flow cytometry to detect A549 and H1299 apoptosis rate; E. Transwell to detect A549 and H1299 migration and invasion capabilities; the values were expressed by mean ± SD (n = 3); versus sh-NC group, * *P* < 0.05.

### 3.3 CircSOX13 acts as a sponge for miR-3194-3p

CircSOX13-regulated downstream genes were explored in this work . Through the bioinformatics website http://starbase.sysu.edu.cn/, it was found that miR-3194-3p had a potential binding site with circSOX13, which might be a circSOX13-regulated downstream gene (Figure 3a). Previous studies have revealed that miR-3194-3p is under-expressed in liver cancer and links with its metastasis and recurrence [19]. This study clarified that miR-3194-3p was under-expressed in NSCLC tissues and cells (Figures 3B and Figure 3C). Additionally, after knocking down circSOX13, miR-3194-3p expression in A549 and H1299 was signally augmented (Figure 3d), revealing that miR-3194-3p was under the regulation of circSOX13. Further DLR experiments revealed that circSOX13-WT reduced the luciferase activity of miR-3194-3p mimic group, whereas circSOX13-MUT had no impact on it (Figure 3e), indicating that circSOX13 acted as a sponge for miR-3194-3p.

**Figure 3.** **CircSOX13 acts as a sponge for miR-3194-3p**. A. Via bioinformatics website http://starbase.sysu.edu.cn/ to query the potential binding sites of miR-3194-3p and circSOX13; B. RT-qPCR to detect miR-3194-3p in NSCLC tissues and normal tissue adjacent to cancer; C. RT-qPCR to detect miR-3194-3p expression in PC9, SPC-A1, H1975, H1299 and A549 and 16HBE; D. RT-qPCR to detect miR-3194-3p expression in A549 and H1299 after transfecting circSOX13-shRNA; E. DLR experiment to detect the targeted binding relationship between miR-3194-3p and circSOX13; the values were mean ± SD (n = 3); versus the normal tissue group, * *P* < 0.05; versus the 16HBE group, ^ *P* < 0.05; versus the sh-NC group, ^#^ *P* < 0.05; versus the mimic NC group, ^&^ *P* < 0.05.

### 3.4 CircSOX13 affects malignant behavior via regulating miR-3194-3p

Next, it was examined whether the malignant behavior of NSCLC regulated by circSOX13 was related to miR-3194-3p. Firstly, the biological functions of miR-3194-3p in NSCLC were examined. The expression of miR-3194-3p in A549 and H1299 cells was up-regulated by transfection with miR-3194-3p mimic (Figure 4a). A series of studies have clarified that elevated miR-3194-3p inhibited the cell viability and proliferation rate, invasion and migration, but promoted apoptosis of A549 and H1299 cells (Figure 4b-Figure 4e).

**Figure 4.** **CircSOX13 influences malignant behavior of NSCLC by regulating miR-3194-3p**. After transfecting miR-3194-3p mimic, A. RT-qPCR to detect miR-3194-3p expression in A549 and H1299 cells; B. CCK-8 to detect A549 and H1299 cell viability; C. Edu analysis to detect A549 and H1299 proliferation; D. Flow cytometry to detect A549 and H1299 apoptosis rate; E. Transwell to detect A549 and H1299 invasion and migration ability; the values were expressed as mean ± SD (n = 3); versus the mimic NC group, * *P* < 0.05.

Subsequently, sh-circSOX13 and miR-3194-3p inhibitor were co-transfected into NSCLC cell lines. As shown in figure 4f, transfection with sh-circSOX13 elevated the expression of miR-3194-3p, which was reversed after co-transfection with miR-3194-3p inhibitor. The studies had manifested that transfection with sh-circSOX13 inhibited A549 and H1299 cell proliferation, invasion and migration, but accelerated apoptosis, which was reversed via co-transfection with miR-3194-3p inhibitor (Figure 4g-Figure 4j). Together, it was suggested that circSOX13 influenced malignant behaviors of NSCLC by regulating miR-3194-3p.

### 3.5 MAPRE1is a target gene of miR-3194-3p

Next, the target genes of miR-3194-3p were given a check. Through the prediction of bioinformatics network, it was found that MAPRE1 had a potential binding site with miR-3194-3p (Figure 5a).MAPRE1 has been proven to be a proto-oncogene [20,21]. We found that MAPREl was highly expressed in NSCLC tissues and cells (Figures 5B and Figure 5C). Additionally, overexpressing miR-3194-3p signally reduced MAPREl levels in A549 and H1299 (Figure 5d), This suggested that MAPRE1 was regulated by miR-3194-3p in NSCLC and might be its downstream target gene. Subsequently, this conjecture was further verified by dual luciferase reporting experiments. And it turned out,MAPRE1-WT could reduce the luciferase activity in miR-3194-3p mimic group, while MAPRE1-MUT had no effect on the luciferase activity in miR-3194-3p mimic group (figure 5f). These findings indicated that MAPREl was highly expressed in NSCLC and was a target gene of miR-3194-3p.

**Figure 5.** **MAPRE1 is the target gene of miR-3194-3p**. A. RT-qPCR to detect MAPRI1 expression in NSCLC tissues and normal tissues adjacent to cancer; B. Western blot to detect MAPRI1 expression in PC9, SPC-A1, H1975, H1299 and A549 and 16HBE C. Western blot to detect MAPRE1 expression in A549 and H1299 cells after transfecting miR-3194-3p mimic; D. Via bioinformatics website http://starbase.sysu.edu.cn/ to query the potential binding sites of miR-3194-3p and MAPRE1; E. DLR experiment to check the targeting relationship between miR-3194-3p and MAPRE1; the values were expressed as mean ± SD (n = 3); versus the normal tissue group, * *P* < 0.05; versus the 16HBE group, ^ *P* < 0.05; versus the mimic NC group, ^#^ *P* < 0.05.

### 3.6 CircSOX13 accelerated malignant behavior of NSCLC via miR-3194-3p/MAPRE1 axis

Later, in our work it was explored whether circSOX13 affected the malignant behavior of NSCLC via regulating miR-3194-3p/MAPRE1 axis. MAPRE1 expression was silenced but overexpressing circSOX13 was manifested, after which circSOX13 and MAPREl levels were elevated signally, but miR-3194-3p level was decreased visually (Figure 6a). Meanwhile MAPRE1 expression was signally reduced after transfecting si-MAPRE1. Later, it was examined the impact of transfection on the biological behavior of NSCLC, finding that overexpressing circSOX13 promoted A549 and H1299 proliferation, invasion and migration but inhibited apoptosis, while simultaneous transfection of si-MAPRE1 reversed them (Figure 6b-Figure 6e). These findings indicated that circSOX13 promoted the malignant behavior of NSCLC via regulating miR-3194-3p/MAPRE1 axis.

**Figure 6.** **CircSOX13 promotes the malignant behavior of NSCLC via miR-3194-3p/MAPRE1 axis**. After transfecting oe-SOX13 and si-MAPRE1, A. RT-qPCR or western blot to detect circSOX13, miR-3194-3p and MAPRI1 expression; B. CCK-8 to detect A549 and H1299 viability; C. Edu analysis to detect A549 and H1299 proliferation; D. Flow cytometry to detect A549 and H1299 apoptosis rate; E. Transwell to detect A549 and H1299 invasion and migration abilities; the values were expressed as mean ± SD (n = 3); versus the oe-NC group, * *P* < 0.05; versus the oe-SOX13 + si-NC group, ^ *P* < 0.05.

### 3.7 CircSOX13 motivates NSCLC Cisplatin resistance

Next, it was examined whether circSOX13 was associated with cisplatin resistance in NSCLC. In order to obtain drug-resistant cell lines, A549 and H1299 cells were treated with different concentrations of DDP and drug-resistant cell lines were named A549/DDP and H1299/DDP cells. As clarified in Figure 7a, IC_50_ values of A549/DDP and H1299/DDP cells were clearly elevated versus parental A549 and H1299 cells, indicating successful induction of the NSCLC drug resistance model. Subsequently, it was examined the expression of circSOX13, miR-3194-3p and MAPRE1 in drug-resistant cell lines and parental cells. The results manifested that the expressions of circSOX13 and MAPRE1 were apparently elevated in A549/DDP and H1299/DDP cells, while the expressions of miR-3194-3p was apparently decreased versus the parental cells (Figure 7b). Subsequently, circSOX13 in A549/DDP and H1299/DDP cells was knocked down (Figure 7c). The results clarified that IC_50_ values of A549/DDP and H1299/DDP cells were distinctly reduced after circSOX13 knockdown (Figure 7d). EDU experiment manifested that knocking down circSOX13 repressed DNA replication of A549/DDP and H1299/DDP cells (Figure 7e). In addition, circSOX13 knockdown apparently reduced the migration and invasion of A549/DDP and H1299/DDP cells, but promoted the apoptosis (figure 7f, Figure 7g). These results suggested that circSOX13 promoted cisplatin resistance in NSCLC.

**Figure 7.** **CircSOX13accelerates NSCLC cisplatin resistance**. A. CCK-8 to detect the IC50 value of A549 and H1299 as well as A549/DDP and H1299/DDP; B. RT-qPCR or western blot to detect circSOX13, MAPRE1 and miR-3194-3p expression in A549 and H1299 and A549/DDP and H1299/DDP; After transfecting circSOX13-shRNA, C. RT-qPCR to detect circSOX13 expression in A549/DDP and H1299/DDP; D. CCK-8 to detect IC_50_ value in A549/DDP and H1299/DDP; E. DNA replication of A549/DDP and H1299/DDP cells detected by Edu analysis; F. Flow cytometry to detect the apoptosis of A549/DDP and H1299/DDP; G. Transwell to detect A549/DDP and H1299/DDP invasion and migration abilities; the values were expressed by mean ± SD (n = 3); versus the A549 group or the sh-NC group, * *P* < 0.05.

### 3.8 CircSOX13 promotes cisplatin resistance in NSCLC via miR-3194-3p/MAPRE1 axis

Next, it was explored whether miR-3194-3p/MAPRE1 axis was involved in the promotion of cisplatin resistance in NSCLC by circSOX13 through functional rescue experiment. Co-transfection of oe-SOX13 and miR-3194-3p mimic was into A549/DDP and H1299/DDP cells. The results clarified that transfection of oe-SOX13 decreased the expression of miR-3194-3p but elevated the expression of MAPRE1, but these effects were prevented by co-transfection of miR-3194-3p mimic (Figure 8a). CCK-8 and Edu experiments (Figure 8b, Figure 8c) showed that transfection of oe-SOX13 increased IC_50_ values and DNA replication of A549/DDP and H1299/DDP cells, but these phenomena were reversed after co-transfection with miR-3194-3p mimic. Flow cytometry manifested that transfection of oe-SOX13 reduced apoptosis of A549/DDP and H1299/DDP cells, but which was recovered by co-transfection of miR-3194-3p mimic (Figure 8d). Transwell clarified that transfection of oe-SOX13 promoted invasion and migration of NSCLC drug-resistant cells, but co-transfection of miR-3194-3p mimic reduced this effect (Figure 8e). These results suggested that circSOX13 promoted cisplatin resistance in NSCLC by regulating miR-3194-3p/MAPRE1 axis.

**Figure 8.** **CircSOX13 promotes cisplatin resistance in NSCLC via miR-3194-3p /MAPRE1 axis**. A. The expression of MAPRE1 and miR-3194-3p in A549/DDP and H1299/DDP cells after co-transfection oe-SOX13 and miR-3194-3p mimic detected by RT-qPCR or Western blot; B. IC_50_ values of A549/DDP and H1299/DDP cells after co-transfection oe-circSOX13 and miR-3194-3p mimic detected by CCK-8; C. DNA replication in A549/DDP and H1299/DDP cells after co-transfection with oe-circSOX13 and miR-3194-3p mimic detected by Edu; D. Apoptosis of A549/DDP and H1299/DDP cells after co-transfection with oe-circSOX13 and miR-3194-3p mimic detected by flow cytometry; E. Transwell to detect the invasion and migration abilities of A549/DDP and H1299/DDP cells after co-transfection with oe-circSOX13 and miR-3194-3p mimic. The values were expressed as mean ± SD (n = 3); versus the oe-NC group, * *P* < 0.05; versus the oe-SOX13 + mimic NC group, ^ *P* < 0.05.

### 3.9 *CircSOX13 promotes tumor growth and cisplatin resistance* in vivo

To support *in vitro* results, it was performed xenotransplantation in nude mice. As shown in Figure 9a-Figures 9c, knocking down circSOX13 or cisplatin treatment reduced tumor volume and weight, while knocking down circsSOX13 at the same time of cisplatin treatment further declined tumor volume and weight. Immunohistochemistry clarified (Figure 9d) that circSOX13 knockdown or cisplatin treatment reduced the number of tumor Ki-67 positive cells, while the combination further inhibited the number of tumor Ki-67 positive cells. Western blot results showed that circSOX13 knockdown and cisplatin treatment reduced MAPRE1 expression separately (Figure 9e). These results manifested that knocking down circSOX13 repressed *in vivo* NSCLC tumor growth and elevated cisplatin sensitivity.

**Figure 9.** **CircSOX13 promotes NSCLC tumor growth and cisplatin resistance**. A. Representative image of tumor; B. Tumor volume; C. Tumor weight; D. Tumor Ki-67 expression detected by immunohistochemistry; E. MAPRE1 protein expression detected by Western blot. The values were expressed as mean ± SD (n = 5); Versus the sh-NC group, * *P* < 0.05; versus the PBS group, ^ *P* < 0.05; versus the DDP + sh-NC group, ^#^ *P* < 0.05.

## 4 Discussion

This work revealed the potential mechanism of a new type of circular RNA circSOX13 in NSCLC development and resistance, finding that circSOX13 is available to promote malignant behavior and cisplatin resistance in NSCLC via sponging miR-3194-3p and up-regulating MAPER1 expression.

Many studies have revealed the role of circRNA in NSCLC. For instance, circ_0017956 promotes NSCLC proliferation and metastasis via regulating miR-515-5p/ITGB8 axis. CircZNF208 enhances NSCLC sensitivity to X-rays rather than carbon ions through miR-7-5p/SNCA signal axis16. Previous studies have reported that circSOX13 is highly expressed in NSCLC tissues. This study further supports such findings In addition, this study showed that circSOX13 was highly expressed in the serum of patients with NSCLC, suggesting that circSOX13 might be a marker for the early diagnosis of NSCLC. However, more clinical analysis (such as ROS curve analysis) are needed to confirm this conjecture. It was in this study also found that circSOX13 promoted the proliferation, invasion, migration but repressed apoptosis of NSCLC, which has been confirmed *in vivo*. Knocking down circSOX13 reduced tumor volume and weight and inhibited the proportion of Ki-67 (a protein highly expressed during cell division) positive cells [22]. These phenomena indicate that circSOX13 is a strong oncogenic gene in NSCLC, and promotes tumor growth of NSCLC by regulating DNA replication and cell division. Cisplatin is an effective tumor-inhibiting chemical drug, but the clinical application of cisplatin has been challenged due to drug resistance of cancer cells [23]. Previous studies have reported the positive effect of inhibiting cisplatin resistance in NSCLC by regulating circRNA, including circASXL1, circPIP5K1A [24], etc. The results of this study suggested that knocking down circSOX13 elevated cisplatin sensitivity in NSCLC *in vivo* and *in vitro*, suggesting that targeting circSOX13 molecules to improve clinical cisplatin resistance has great potential later.

Recently, a study reported that 22 tumor-derived miRNAs are differentially expressed in NSCLC patients and healthy people [25]. Increasing studies have revealed the relationship between miRNA and NSCLC malignant phenotype and resistance. Cui D *et al*. found that miR-138-5p improves NSCLC proliferation, invasion and migration via regulating epidermal growth factor receptor and PI3K/Akt signaling [26]. Additionally, miR-638 is available to inhibit NSCLC development via repressingFOSL2 expression [27]. Amid exploring the resistance mechanism, the researchers found that miR-139-5p [28], miR-1/133a, miR-206/133b cluster [29], and miR-221-3p23 promotes NSCLC sensitivity to chemical drugs which include cisplatin, gefitinib, osimertinib, paclitaxel and so on. Here, it was probed into the effect of miR-3194-3p on NSCLC malignant phenotype and cisplatin resistance, finding that miR-3194-3p is lowered in NSCLC, which restrainsNSCLC proliferation, migration and invasion but promotes its apoptosis. Additionally, cisplatin is available to reduce miR-3194-3p expression in NSCLC, and it participates in the regulation of circSOX13 on cisplatin resistance in NSCLC. This supports the previous report that miR-3194-3p inhibits the breast cancer [30] and hepatocellular carcinoma.

Next, in this work it was further exploited the potential gene effectors participating in the biological functions of NSCLC. Through bioinformatics screening and dual luciferase verification, it was found that MAPREl is the target gene of miR-3194-3p and is regulated by circSOX13. As a proto-oncogene, MAPRE1 has been proved to be highly expressed in nasopharyngeal carcinoma, liver cancer, colorectal cancer [31], gastric cancer [32] and others. It can be applied as a diagnostic biomarker and links with poor prognosis. This study found that silencing MAPRE1 reversed the role circSOX13 played in promoting NSCLC, indicating that MAPRE1 also acts as a proto-oncogene in NSCLC. In addition, in this study the important role of MAPRE1 is firstly revealed in cisplatin resistance in NSCLC. The expression of MAPRE1 is up-regulated after cisplatin treatment, and circSOX13 elevates cisplatin resistance by promoting MAPRE1 in cisplatin resistant NSCLC cell lines and tumors.

## 5 Conclusion

In conclusion, our findings indicate that circSOX13 is highly expressed in NSCLC, and it is available to promote the malignant behavior and cisplatin resistance in NSCLC via competitive bindingmiR-3194-3p to mediate MAPREl expression. This provides a new target for improving the survival rate and resistance in NSCLC later. But the role of circSOX13 in NSCLC *in vivo* needs further study.
